# Is Refracture a Concern Following Closed Management of Tibia Shaft Fractures in Children?

This article has been retracted.

**DOI:** 10.7759/cureus.7206

**Published:** 2020-03-08

**Authors:** Eli Ahdoot, Ryne Jenkins, Theresa Pak, Henry Tsang, Juston Fan

**Affiliations:** 1 Orthopaedic Surgery, Riverside University Health System Medical Center, Moreno Valley, USA; 2 Orthopaedic Surgery, Riverside University Health System Medical Center, Moreno Valley , USA

**Keywords:** pediatric fractures, refracture, tibia shaft fracture, conservative management

## Abstract

Purpose: Tibia shaft fractures account for 15% of all pediatric fractures. These fractures are often treated nonoperatively with closed reduction and long leg casting. In children treated nonoperatively, refracture can cause significant frustration to both the patient and their family in addition to a delay in resuming normal activities for several months. The purpose of this study was to investigate the rate of refracture of tibia shaft fractures treated nonoperatively at our institution.

Methods: We performed a retrospective chart review of pediatric patients at one institution with the diagnosis of a tibia shaft fracture who were treated nonoperatively between January 1, 2000 and December 31, 2016. Exclusion criteria included those without complete retrievable radiographs or without radiographic confirmation of healed fracture. Patients who sustained a proximal or distal metaphysical tibia fracture or a toddler fracture were also excluded. Additionally, those with less than three months of clinic follow-up or an underlying metabolic bone disease were excluded. Data such as age, sex, body mass index, mechanism of injury, location of fracture, initial displacement, angulation, treatment, length of immobilization, and complications were recorded. The primary outcome for our study was the presence of refracture. Refracture was defined as a repeat fracture of the tibia at the same location within 18 months of the original fracture.

Results: A total of 64 patients met the inclusion criteria and were included in the study. Of the 64 patients, only one patient sustained a refracture. The refracture occurred eight months after the initial injury and required operative intervention. This rate of refracture is equated to roughly 1.5%.

Conclusion: Conservative management of closed tibia shaft fractures with casting is an ideal treatment for pediatric fractures. Conservative management allows for avoidance of surgical intervention and low refracture rates. This study provides support regarding the adequacy of conservative management with limited complications. Although the rate of refracture still exists, patients and families should be counseled that the rate of healing without complications is about 98.5%.

## Introduction

Pediatric tibia fractures account for 15% of all pediatric fractures [1]. These include both traumatic injuries and toddler’s fractures, defined as ambulatory children aged nine months to three years who have sustained a low-energy spiral fracture of their tibia [2]. Tibia fractures are common and are predominantly treated nonoperatively with long leg casting [3]. These fractures typically heal without sequela and within six to twelve weeks [3]. However, certain indications require operative management of tibia fractures. Such circumstances make up less than 5% of tibia fracture cases and include open fractures, multiple long bone fractures, unacceptable alignment after closed reduction (>10° of angulation, >1 cm shortening), neurovascular injury, and compartment syndrome [3]. In those patients treated nonoperatively, refracture can cause significant frustration to both patient and family. Additionally, patients experience an additional delay in activities for several months to follow. Refracture in pediatric upper extremity fractures has been shown with rates ranging from 1% to 8%; however, there is limited literature regarding refracture rates in pediatric tibial shaft fractures [4,5]. The purpose of this study is to identify the rate of refracture at our institution and any possible modifiable risk factors. Thus, we may be able to adjust treatment guidelines ultimately decreasing the incidence of refracture and allowing children to return back to play at an earlier time frame.

## Materials and methods

Study design, setting, and population

We performed a retrospective chart review of pediatric patients treated nonoperatively with the diagnosis of a tibia shaft fracture between January 1, 2000 and December 31, 2016. Patients with ages ranging three to sixteen years were included in the study. Three months of follow-up or radiographs demonstrating healing at final follow-up prior to three months were required. Patients with less than three months of follow-up and without radiographic confirmation of healed fracture were excluded. Patients who sustained a proximal or distal metaphyseal tibia fracture or a toddler fracture were also excluded. Additionally, those with underlying metabolic bone disease or those without complete retrievable radiographs were excluded. Data were obtained from emergency room consultations and clinic notes.

Standard protocol approvals, registrations, and patient consents

This study was performed with approval of the Children’s Hospital of Orange County Institutional Review Board.

Data collection

Basic patient and hospital demographics were recorded including age, sex, date of injury, body mass index, mechanism of injury, location of fracture, initial displacement, angulation, type of fracture, treatment, length of immobilization, refracture date of injury, refracture mechanism, refracture treatment, and complications. Refracture was defined as having a fracture at the same site of initial injury within 18 months of the first fracture [4]. The primary outcome for our study was the rate of refracture.

Treatment protocol

Initial treatment at our institution includes long leg casting with or without manipulation. Patients are placed in a long leg cast for a minimum of four weeks. Serial radiographs are completed at clinic visits weekly or biweekly depending on severity to monitor for healing, neurovascular changes and potential deformities. Patients are then transitioned to weight bearing as tolerated in a short leg cast for an additional four weeks.

## Results

Between 2000 and 2016, there were 64 patients meeting the study criteria (see Figure 1). A total of 43 (64%) patients sustained a midshaft tibia fracture and 21 (33%) patients sustained a distal tibia fracture. One patient in the midshaft tibia group sustained a refracture. The refracture occurred eight months after the initial injury and required operative intervention. This rate equated to roughly 1.5%. Radiographic evidence of healing was seen in two to eighteen months. Because there was only one refracture, we were not able to identify risk factors that may correlate with an increased refracture rate.

**Figure 1:** Cohort Ascertainment Flowchart describing the ascertainment of patients with tibial shaft fractures.

## Discussion

Conservative management of closed, displaced tibia fractures with reduction and casting is an appropriate treatment for pediatric fractures that allows for avoidance of surgical intervention and associated complications. This study provided scientific support, of which there is minimal, regarding the benefits of conservative management in pediatric tibia fractures. The results of our study provide reassurance that conservative treatment is adequate with a minimal refracture rate and associated outcomes. When weighing treatment options, age is an important factor of what is acceptable and what is tolerable. Younger children are able to tolerate nonanatomic reductions because of their ability for bony growth. However, adolescents have been shown to have a 40% failure rate with closed reduction [4]. Our study showed radiographic evidence of healing ranging from two to eighteen months. Prior studies have shown time to fracture healing varies according to age with children ranging from four to six weeks and adolescents ranging from eight to twelve weeks [6].

Close monitoring of fracture healing is essential for a favorable outcome with leg casting. Loss of reduction can occur secondary to atrophy and resolution of swelling [6]. Additionally, physical loads and traction from muscles can alter fracture alignment as patients begin to weight-bear. Isolated tibial shaft fractures with intact fibulas can shorten and form a varus misalignment secondary to forces on the distal tibia from the posterior compartment muscles [6]. Fractures with both tibia and fibula involvement can shorten and form a valgus misalignment as forces are applied distally by the muscles of the lateral and anterior compartments.

Interestingly, a 2012 comparison of 80 pediatric patients treated with long leg casting showed immobilization with the knee flexed to 10 degrees and immediate weight bearing as tolerated had no significant difference in the time to union, fracture angulation, and shortening at the fracture site as compared to patients immobilized at 60 degrees of flexion and instructed not to weight-bear [7]. Future studies are needed; however, patients may be able to further benefit from conservative management if allowed to weight-bear early on in recovery.

Although our study did review several patient fracture factors, we were unable to assess identifiable risk factors of refracture because there was only one refracture in our study. The rate of refracture still exists; however, patients and families should be counseled that the rate of healing is about 98.5% with conservative management. Reassurance should be provided, and patience should be emphasized as the healing process takes several months for children to return to their full activity level with previous studies showing an average of 15 weeks [8].

## Conclusions

This is the first study to discuss tibia refracture rates in the pediatric population. The study also reveals that there is a safe and predictable role in conservative management in tibia shaft fractures with a refracture rate of 1.5%. With this knowledge, patients and families should be reassured of the high success rate and ability to avoid possible complications and costs related to surgical management.
